# Comparative Studies on a Standardized Subfraction of Red Onion Peel Ethanolic Extract (Plant Substance), Quercetin (Pure Compound), and Their Cell Mechanism and Metabolism on MDA-MB-231

**DOI:** 10.1155/2022/9284063

**Published:** 2022-09-07

**Authors:** Kar Xin Leong, Sin Pei Chao, Poh Chiew Siah, Shern Kwok Lim, Boon Yin Khoo

**Affiliations:** Institute for Research in Molecular Medicine (INFORMM), Universiti Sains Malaysia (USM), Penang, Malaysia

## Abstract

This study indicates the presence of quercetin in subfraction F1 and the standardized value of F1 derived from research using ultra-performance liquid chromatography (UPLC) and AlCl_3_ colorimetric assays, which further proved that both F1 and quercetin are potential growth inhibitors in MDA-MB-231 cells by 3-(4,5-dimethylthiazol-2-yl)-2,5-diphenyltetrazolium bromide (MTT) assay. In the process, staining of F1-treated cells with annexin/propidium iodide (PI) reduced cell proliferation and induced only S and G2 phases of cell cycle arrest in the treated cells by flow cytometry. Quercetin reduced cell proliferation by inducing apoptosis and S phase arrest. The 5′-bromo-2′-deoxyuridine (BrdU) incorporation of DNA synthesis in MDA-MB-231 cells was also inhibited after F1 and quercetin treatments. F1 and quercetin induced CYP1A1 and CYP1B1 gene expression, but only F1 induced CYP2S1 gene expression in the treated cells. Both F1 and quercetin inhibited the proliferation of MDA-MB-231 cells in different ways, but F1 is likely a better potential anticancer agent derived from the green approach towards breast cancer treatment.

## 1. Introduction

Phytochemicals stimulate physiological pathways, which may be beneficial for modulating cancer development [1–5]. Therefore, more studies on natural products or compounds to explore the anticancer properties for alternative cancer therapeutics with reduced toxicity are warranted. Red onion is rich in bioactive compounds and displays numerous pharmacological properties, including antimicrobial, antioxidant, anti-inflammatory, antihypertensive, and immunoprotective effects. Considerable epidemiological research has also revealed that this vegetable exhibits anticancer therapeutic value [6–9], and dietary intake of onion has been shown to reduce the risk of developing breast cancer [10, 11]. Therefore, the potential of natural products derived from onions containing these highly bioactive compounds could be used as new anticancer agents. A closer inspection of several alternative medical treatments has also proven that onion-derived natural products carry anticarcinogenic properties with less toxicity.

This study aimed to indicate the presence of quercetin (the main flavonoid of red onion peel ethanolic extract) in a subfraction of red onion peel ethanolic extract (F1) and the standardized value of F1 derived from research using ultra-performance liquid chromatography (UPLC) and aluminium chloride (AlCl_3_) colorimetric assays. The study then investigated the growth inhibitory effect of F1 and quercetin. The analysis used red onion peel instead of flesh because the peel contains higher concentrations of quercetin aglycon than the flesh [12, 13]. The F1 produced in-house contains high quercetin levels that can be considered a potential anticancer agent. Preliminary results showed that F1 reduced the growth of breast cancer MCF-7 cells. The study also showed a better *in vitro* anticancer effect for F1 than for camptothecin (a commercially used anticancer drug) on oral cancer CAL-27 cells. Many *in vitro* and *in vivo* studies have also been conducted to confirm the anticancer properties of red onion peels. However, the cellular mechanism and cell metabolism induced by F1 have not been studied in detail. This study first investigated the phytochemical properties of F1 and the cytotoxic effects of both F1 and quercetin in MDA-MB-231 cells. Then, the study examined the cell cycle profile, apoptosis induction, and 5′-bromo-2′-deoxyuridine (BrdU) incorporation of DNA synthesis in MDA-MB-231 cells. The mRNA expression of CYP genes in F1- and quercetin-treated MDA-MB-231 cells was also investigated in this study. The findings will facilitate the discovery of a green approach to novel anticancer agents from natural products for breast cancer treatment with bioavailable, safe, cost-effective, and minimal side effect properties in the future.

## 2. Materials and Methods

### 2.1. Determination of Total Flavonoid and Quercetin Content by UPLC and AlCl3 Colorimetric Assays

Quercetin content in subfraction F1 was detected by an ACQUITY UPLC system (Waters Corporation, Milford, MA, USA) incorporated with a photodiode array as the detector in the School of Biological Sciences, USM. F1 was prepared as described in Chao's previous study [14]. A 2.0 *μ*L aliquot of F1 or quercetin standard solution was injected into the UPLC BEH C18 column (100 mm × 2.1 mm i.d., 1.7 *µ*m particle size, Waters Corporation, Milford, Massachusetts, USA). The standard and sample solutions were injected twice to ensure reproducibility. The temperature was set at room temperature, and the mobile phase used was isocratic mode, in which elution was performed with 95% acetonitrile. The flow rate of the analysis was set as 0.1 mL/min with a total runtime of 10 min (7 min for analysis and 3 min reequilibration). The detection of the elution peaks was set at *λ* = 360 nm. The retention time shown in the chromatograms by Empower 2 Software (Waters Corporation, Milford, MA, USA) indicated the presence and the level of quercetin in the F1 solution. The total flavonoid content in F1 was also determined by an AlCl_3_ colorimetric assay adapted from Sembiring's study [15] with slight modification. First, 50 *μ*L F1 (1.0 mg/mL) and various concentrations of quercetin standard solution (25, 50, 100, and 200 *μ*g/mL) were prepared. Absolute ethanol was used instead of quercetin or sample solution as the blank solution. Each solution was then added to the respective well in the 96-well plate. Then, 150 *μ*L of 99.7% ethanol and 10 *μ*L of 10% (w/v) AlCl_3_ solution were added to each well. Next, 10 *μ*L of 1.0M sodium acetate solution was added to the solution mixture in the wells. All reagents in the wells were mixed and incubated for 40 min at room temperature in the dark. The absorbance of the standard versus blank solutions was then quantified at 415 nm using a Multiskan Spectrum Microplate Reader (Thermo Fisher Scientific, Waltham, MA, USA). The absorbance of the sample and standard solutions was also measured in a range of wavelengths from 350 to 600 nm using a microplate reader for purity analysis. All sample and standard solutions were prepared in triplicate, and the absorbance values were measured, recorded, and interpolated into the linear quercetin calibration curve. The linear regression equation of the calibration curve for a straight line is *Y* = *mx* + *c*, where *Y* = absorbance of extract, *m* = slope of the calibration curve, *x* = concentration of F1, and *c* = intercept. The total flavonoid content of F1 was expressed as mg quercetin equivalents (QEs) per gram of dry extract (mg/g) and calculated by using the following formula: C = cV/M, where C = total flavonoid content of F1 (mg QEs/g dry extract), *c* = concentration of quercetin obtained from the calibration curve in mg/mL, V = volume of extract in mL, and M = mass of extract in grams.

### 2.2. Breast Cancer Cell Culture, Seeding, and Treatment

The MDA-MB-231 (ATCC®HTB-26™) cell line was purchased from the American Type Culture Collection (ATCC, VA, USA). The cells were cultured in complete growth medium in T-25 or T-75 tissue culture flasks (Nunc, Roskilde, Denmark). The growth medium contained high glucose Dulbecco's Modified Eagle's Medium (DMEM; Thermo Fisher Scientific, Inc.) supplemented with 10% (v/v) fetal bovine serum (FBS; Thermo Fisher Scientific Inc.), 100 units/mL penicillin, and 100 *µ*g/mL streptomycin. The MDA-MB-231 cells were incubated at 37°C in a humidified atmosphere of 5% (v/v) carbon dioxide (CO_2_) and grown with a doubling time of approximately 38 h. The MDA-MB-231 cells were trypsinized when the number of cells in the culture flasks had reached sufficient growth. The cells were seeded in 96-well plates at a cell density of 2 × 10^4^ cells/mL for growth inhibitory effect analysis or in 6-well plates at a cell density of 1.2 × 10^6^ cells/mL for cell cycle, apoptotic effect, DNA synthesis, and CYP mRNA expression analyses. The cells were then subjected to treatment with 0.1% dimethyl sulfoxide (DMSO) (control), 50 *μ*g/mL F1 (determined in this study), or 60 *μ*g/mL quercetin [16] in growth media that contained only 2% FBS. The treated cells were incubated at 37°C in a 5% (v/v) CO_2_ incubator for 24, 48, and 72 h prior to further analysis.

### 2.3. Growth Inhibitory Effect Analysis of F1 and Quercetin by MTT Assay

The cells treated with F1 and quercetin in 96-well plates, as described above, at the end of each incubation period were added to 24 *μ*L of 5 mg/mL MTT reagent (Sigma-Aldrich, St. Louis, MO, USA) in each well. The reaction was incubated for 4 h. The solution was carefully removed without disturbing the formazan crystals formed in each well. Next, 100 *μ*L acidified isopropanol (Sigma-Aldrich, St. Louis, MO, USA) was added to each well and agitated to promote homogeneous colour development. Following colour development, the colour intensity in each well was read at 570 nm using an enzyme-linked immunoassay (ELISA) plate reader (Tecan, Männedorf, Switzerland).

### 2.4. Cell Cycle Analysis of F1- and Quercetin-Treated MDA-MB-231 Cells by Flow Cytometry

The cells treated with F1 and quercetin in 6-well plates, as described above, were trypsinized at the end of each incubation period, and the cell suspension was transferred into Falcon tubes. The cell suspension with the old medium in the tube was centrifuged at 1,000 g for 5 min. The supernatant was then discarded, and the cell pellet was washed with phosphate-buffered saline (PBS). After washing, a 1 × 10^6^ cell suspension was transferred into new Falcon tubes, and the cell suspension was then centrifuged as above. The cells were then fixed and permeabilized by adding 70% ice-cold absolute ethanol dropwise with gentle mixing. The cell suspension was then stored at 4°C overnight to allow fixation. The ethanol-fixed cells were centrifuged at 1,000 g for 10 min and washed by resuspending the cells in PBS. The washed cells were then stained with 500 *μ*L FxCycle™ propidium iodide (PI)/RNAse Staining Solution (Thermo Fisher Scientific, MA, USA) in the dark for 30 min. The stained samples were transferred into new sterile flow tubes and kept on ice until they are subjected to flow cytometry analysis using a BD FACSCalibur (BD Biosciences, NJ, USA). Cell cycle distribution was analyzed from a total of 15,000 events with CellQuest software 3.3 (BD Biosciences, New Jersey, USA). The percentage of cells in each phase was analyzed and plotted as a DNA histogram using ModFit LT™ software (BD Biosciences, NJ, USA). The entire analysis was performed at the Advanced Medical and Dental Institute (AMDI), USM in Bertam, Penang.

### 2.5. Apoptotic Effect Analysis of F1- and Quercetin-Treated MDA-MB-231 Cells by Flow Cytometry

The cells treated with F1 and quercetin in 6-well plates, as described above, were also subjected to apoptotic effect analysis using the annexin V-fluorescein isothiocyanate (FITC) apoptosis detection kit (Thermo Fisher Scientific, MA, USA). Briefly, the trypsinized cells collected in 15 mL Falcon tubes were centrifuged at 400 g for 4 min at 4°C to remove the old medium. Then, the cells were washed twice with 3 mL cold PBS. The cell suspension was counted, and 5 × 10^5^ cells/mL were transferred into new Falcon tubes. The cells were centrifuged to remove the supernatant, and then the cell pellet was resuspended in 200 *μ*L of 1*x* binding buffer. A volume of 5 *μ*L annexin V-FITC was then added to 195 *μ*L of the cell suspension, mixed well, and incubated in the dark at room temperature for 10 min. The cells were then washed with 200 *μ*L of 1*x* binding buffer. The cells were resuspended in 190 *μ*L of 1*x* binding buffer prior to the addition of 10 *µ*L of 20 *μ*g/mL PI. The mixture was transferred to a new sterile tube for flow cytometry analysis using a BD FACSCalibur (BD Biosciences, NJ, USA) with 488 nm excitation, 655–730 nm emission for PI, and 525 nm emission for FITC.

### 2.6. DNA Synthesis Analysis of F1- and Quercetin-Treated MDA-MB-231 Cells by BrdU

The cells treated with F1 in 6-well plates were also subjected to incorporation of 1.0 mM BrdU labelling solution (BrdU; Invitrogen, Thermo Fisher Scientific, Waltham, MA, USA) into newly synthesized DNA (surviving mitosis ability) in the dark. The cells were then washed, trypsinized, and counted, whereby 1.0 × 10^6^ cells of cell suspension from each treatment were pipetted into a 15 mL Falcon tube. The BrdU-labelled cells were incubated before the cells were spun down at 1,000 g for 5 min. The BrdU-labelled cells were then fixed and permeabilized with 5 mL fixation dropwise. The cell suspension was then stored at −20°C overnight to allow fixation, and then the cells were subjected to washing steps. The steps of DNA denaturation, neutralization of the acidic treatment, and finally resuspension of the cell pellets with the antibody staining solution were performed. The cell suspensions were then added to the anti-BrdU monoclonal antibody conjugated with FITC. The stained cells were then incubated and washed again, as described above, and resuspended in 500 *μ*L PBS. The cell suspensions were then stained with 500 *μ*L FxCycle™ PI/RNase Staining Solution. The stained cells were collected, as described above, and then transferred into a 5 mL round bottom polystyrene test tube. The tube was placed on ice prior to analysis with flow cytometer analysis using CellQuest software version 3.3 (BD Biosciences, Franklin Lakes, NJ, USA) from a total of 15,000 events. The percentage of BrdU-positive cells was analyzed using Summit software version 1.4 (Beckman Coulter, Brea, CA, USA).

### 2.7. CYP Expression Analysis in F1- and Quercetin-Treated MDA-MB-231 Cells by Real-Time PCR

The cells treated with F1 and quercetin in 6-well plates, as described above, were also subjected to total RNA extraction using TRIzol Total RNA Isolation Reagent (Life Technologies Corporation, Carlsbad, CA, USA). The extracted total RNA pellet was then air-dried for 15 min and resuspended in 25 *μ*L RNase-free water. Only the extracted total RNA with an absorbance A260/A230 ratio within 1.8–2.0 and an A60/280 ratio within 2.0–2.2, assessed using a NanoDrop™ 2000C spectrophotometer (Thermo Fisher Scientific, USA), was used for cDNA conversion. The bands that indicated a good quality of RNA, assessed by 1% (w/v) agarose gel electrophoresis, were visualized and captured under UV light by an image analyzer (Syngene, Cambridge, UK). The extracted total RNA was then reverse-transcribed to cDNA using a Tetro cDNA Synthesis Kit (Bioline, London, UK). The reverse transcription products (cDNA) were kept at −20°C until the products were used for real-time polymerase chain reaction (PCR) gene expression analysis. All primers were designed using Primer Express software v3.0.1 (Thermo Fisher Scientific, Massachusetts. USA; Table 1). All oligonucleotide primers ordered from Integrated DNA Technologies (Coralville, USA) were packed in desalted lyophilized form. The primer stocks were dissolved in RNase-free water (Sigma-Aldrich, St. Louis, MO, USA) to generate a final 100 *µ*M concentration of each primer solution. The primer solutions were stored at −20°C until use. Real-time (RT) PCR was performed using an Agilent AriaMx Real-Time PCR System (Agilent, California, USA). The PCR cocktail was prepared by adding 10 *µ*L iTaq™ Universal SYBR Green Supermix (Bio-Rad, CA, USA), 0.8 *μ*L of 10 *μ*M forwards, and reverse primers, each for the gene of interest (GOI), and 50 ng cDNA diluted in nuclease-free water to a total volume of 20 *μ*L in each well of 0.1 mL, 8-tube quantitative (q) PCR strips (AITbiotech, Singapore). The reactions were initiated with a hot start at 95°C for 30 sec, followed by 40 cycles of amplification at 95°C for 15 sec as the denaturation step and 60°C for 1 min as the annealing and extension step. The reactions were continued at 1 cycle of thermal profile consisting of 95°C for 15 sec, followed by 60°C for 1 min, 95°C for 30 sec, and 60°C for 15 sec to generate a melting curve. The expression value of GOI was normalized to glyceraldehyde-3-phosphate dehydrogenase (GAPDH), whereby the relation between the normalized GOI in treated and vehicle control samples was determined by the fold change using the 2^−ΔΔCt^ method [17]. The fold change value for the vehicle control was set as 1, whereas an expression change value >1 represented upregulation, and a value of <1 represented downregulation of the gene.

### 2.8. Statistical Analysis

GraphPad Prism version 8.2.1 for Windows (GraphPad Software Inc., La Jolla, CA, USA) was used to generate the dose-response growth curves. The statistical analysis is presented as the mean ± standard deviation (SD) of triplicate determinations. One-way analysis of variance (ANOVA) was used to analyze the mRNA gene expression with an additional Dunnett's multiple comparisons test to compare 2 among 3 or more datasets. Data analysis was also performed for photographs using ImageJ scientific program (National Institutes of Health). The level of significance was set at *α* = 0.05 (95% confidence interval), where the confidence levels were indicated as statistically significant by asterisks *∗* for *p* values <0.05, *∗∗* for *p* values <0.01, and *∗∗∗* for *p* values <0.001.

## 3. Results

### 3.1. Total Flavonoid Content of F1

The analysis of total flavonoid and quercetin content in subfraction F1 using UPLC shows a narrow, sharp peak at approximately 2.5 min with a slight shoulder peak towards the right side of the chromatogram. The retention time of F1 (1,000 *μ*g/mL) falls at approximately 2.549 to 2.553 min (Figures 1(a) and 1(b)), whereas the analysis detected 200 µg/mL quercetin at a retention time of 2.566 min (Figure 1(c)). UPLC analysis showed that the retention time of F1 was similar to the retention time of quercetin. The analysis predicted the quercetin content of F1 to be approximately 135.085 *μ*g/mL. The AlCl_3_ colorimetric assay further revealed that the total flavonoid content in F1 was approximately 193.07 to 200.63 mg of quercetin equivalent (QE) per gram of dry extract (mg/g) using a standard curve (Figure 1(d)). F1 contains a high concentration of flavonol compounds, such as quercetin and its derivatives. The purity analysis showed a similar absorbance pattern at an absorbance peak of 420 nm, identical to the absorbance peak recorded for quercetin (data not shown). This result supports the presence of quercetin in F1 and the standardized value of F1 derived from our research.

### 3.2. Cytotoxic Effects of F1- and Quercetin-Treated MDA-MB-231 Cells

The cytotoxic effect of F1 in MDA-MB-231 cells resulted in the ideal dose-response of the test compound on the cancer cells at 24 h (hillslope = −0.49; maximal response ≤25%) (Figure 2(a)) and 48 h (hillslope = −0.76; maximal response ≤25%) of treatment (Figure 2(b)). However, the ideal dose-response of F1 on the cancer cells did not persist until 72 h of treatment (Figure 2(c)). The ideal dose-response of quercetin was not observed on the cancer cells at 24 h of treatment (Figure 2(d)). The ideal dose-response of quercetin was observed on the cancer cells only at 48 h (hillslope = −2.247; maximal response ≤75%) (Figure 2(e)) and 72 h (hillslope = −2.785; maximal response ≤50%) of treatment (Figure 2(f)). Although quercetin showed a good later growth inhibitory effect on the cancer cells following 72 h of treatment, F1 showed a good early growth inhibitory effect on MDA-MB-231 cells. For the half-maximal effective concentration (EC_50_) value, only MDA-MB-231 cells after F1 treatment for 48 h showed an EC_50_ value ≤50 *μ*g/mL (10.22 *μ*g/mL); compounds that exhibited an EC_50_ value ≥50 *μ*g/mL were considered inactive. The differences in growth inhibitory activity of F1 and quercetin indicate that F1 is better suited for treatments that require immediate effect, while quercetin can be used for long-term treatment.

### 3.3. Cell Cycle Profile of F1- and Quercetin-Treated MDA-MB-231 Cells

The histograms of the cell cycle profile of MDA-MB-231 cells treated with 0.1% DMSO (control), 50 *μ*g/mL F1, and 60 *μ*g/mL quercetin for 24, 48, and 72 h showed changes in the phases of the cell cycle (Figure 3(a)). The cell population in S phase for F1-treated MDA-MB-231 cells increased significantly to 53.13% (*p* < 0.001), accompanied by a decrease in the cell population in the G0/G1 phase to 39.68% (*p* < 0.001), compared to the respective controls (DMSO-treated MDA-MB-231), but with no significant effect on the cell population in G2/M phase at 24 h of treatment (Figure 3(b) (A)). Conversely, the distribution of cell cycle phases in MDA-MB-231 cells treated with quercetin for 24 h showed no significant difference compared to the controls. At 48 h of treatment, a significant increase in the cell population in both the S phase (39.34%; *p* < 0.001) and G2/M phase (39.70%; *p* < 0.001) was observed in F1-treated MDA-MB-231 cells, where a drop in the cell population to only 20.96% (*p* < 0.001) was observed in the G0/G1 phase compared with the controls (Figure 3(b) (B)). Quercetin only caused a reduction in the cell population in G0/G1 phase to 70.53% (*p* < 0.001) and an increase in the cell population in S phase to 25.72% (*p* < 0.001), but it had no significant effect on the cell population in G2/M phase. At 72 h of treatment, F1-treated MDA-MB-231 cells showed a further reduced cell distribution in the G0/G1 phase (27.09%, *p* < 0.001) with increased distribution in both the S (31.52%, *p* < 0.001) and G2/M (41.39%, *p* < 0.001) phases at 72 h of treatment (Figure 3(b) (C)). Similarly, quercetin-treated MDA-MB-231 constantly underwent cell cycle progression, shifting only from G0/G1 phase (61.02%, *p* < 0.001) to S phase (36.88%, *p* < 0.001) with no effect on the G2/M phase. This phenomenon implies that F1 induced cell cycle arrest at both the S and G2/M phases, but quercetin induced cell cycle arrest at the S phase only in MDA-MB-231 cells.

### 3.4. Apoptosis Induction of F1- and Quercetin-Treated MDA-MB-231 Cells

Histograms of the cell death effect of MDA-MB-231 cells treated with 0.1% DMSO (control), 50 *µ*g/mL F1, and 60 *µ*g/mL quercetin for 24, 48, and 72 h are shown in Figure 4(a). Analysis of the effect revealed that F1 did not induce apoptosis in MDA-MB-231 cells after 72 h of treatment compared to the controls (DMSO-treated MDA-MB-231), but apoptosis was induced in quercetin-treated MDA-MB-231 cells. There was a significant increase in the cell population at the early and late apoptosis stages, as indicated by an increase in the cell population from 2.99% in the control to 6.61% (*p* < 0.001) and from 2.69% in the control to 3.36% (*p* < 0.05), respectively, in quercetin-treated MDA-MB-231 cells at 24 h of treatment (Figure 4(b) (A)). When quercetin treatment was prolonged to 48 h, 7.71% (*p* < 0.001) and 5.26% (*p* < 0.001) of cells were observed in the early and late apoptosis stages, respectively, compared to 2.43% of the control in the early apoptosis stage and 2.42% of the control in the later apoptosis stage (Figure 4(b) (B)). The apoptotic effect induced by quercetin at 72 h of treatment was most significant, as 18.48% (*p* < 0.001) was found in the early apoptosis stage and 8.13% (*p* < 0.001) in the late apoptosis stage (Figure 4(b) (C)). A significant reduction in cell viability from 90.96% in the control to 70.95% (*p* < 0.05) in the quercetin-treated MDA-MB-231 cells was also observed after 72 h of treatment, suggesting that quercetin could induce apoptosis in MDA-MB-231 cells but F1 did not (data not shown).

### 3.5. DNA Synthesis of F1-Treated MDA-MB-231 Cells

The histograms of the proportion of BrdU-positive MDA-MB-231 cells treated with 0.1% DMSO (control), 50 *µ*g/mL F1, and 60 *µ*g/mL quercetin for 24, 48, and 72 h (Figure 5(a)) represent the total DNA content of the cell population in various stages of the cell cycle. The dot-plot analysis showed that the percentage of BrdU-positive MDA-MB-231 cells treated with 50 *µ*g/mL F1 and 60 *µ*g/mL quercetin was higher than that of BrdU-positive MDA-MB-231 cells in control after 24 and 48 h of treatment (Figure 5(b)). MDA-MB-231 cells treated with 50 *µ*g/mL F1 showed a slight reduction in the percentage of BrdU-positive cells after F1 treatment for 24 h (49.54%; *p* < 0.01) and 48 h (46.17%; *p* < 0.05), but the percentage of positive cells remained high. A remarkable increase in the percentage of BrdU-positive MDA-MB-231 cells was observed after treatment with 60 *µ*g/mL quercetin for 24 h (57.74%; *p* < 0.001) and 48 h (54.93%; *p* < 0.01). The MDA-MB-231 cells treated with F1 showed a similar percentage (39.16%) of BrdU-positive cells to the control (36.25%) after 72 h of treatment. The analysis also showed a reduction in the percentage of BrdU-positive cells in MDA-MB-231 cells treated with quercetin (31.48%) compared to the control (36.25%) after 72 h of treatment, although it was not significant. The BrdU-positive cells that incorporated the DNA of dividing cells during the S phase of the cell cycle could still be observed after 24 and 48 h of F1 and quercetin treatments. This phenomenon demonstrated that DNA synthesis is not fully inhibited by 50 *µ*g/mL F1 and 60 *µ*g/mL quercetin in MDA-MB-231 cells at 24 and 48 h of treatment.

### 3.6. mRNA Expression of CYP Genes in F1- and Quercetin-Treated MDA-MB-231 Cells

The analysis observed the optimum level of CYP1A1 mRNA expression at 48 h of treatment compared with the control (DMSO-treated MDA-MB-231), where the level of CYP1A1 was upregulated to a much lower extent in F1-treated MDA-MB-231 cells than in quercetin-treated MDA-MB-231 cells (Figure 6(a)). The mRNA expression of CYP1A1 in F1- and quercetin-treated cells had 6.8-fold (*p* < 0.01) and 20.8-fold (*p* < 0.001) upregulation, respectively, compared with the control at 48 h of treatment. Then, only CYP1A1 mRNA expression in quercetin-treated cells remained upregulated by a 13.2-fold change (*p* < 0.001) for 72 h of treatment. Both F1 and quercetin also showed a similar optimum profile of CYP1B1 mRNA expression, with 3.15-fold (*p* < 0.05) and 4.60-fold (*p* < 0.01) changes, respectively, in MDA-MB-231 cells after 48 h of treatment (Figure 6(b)). The results further showed significant upregulation of CYP1B1 mRNA expression following 72 h of quercetin treatment in MDA-MB-231 cells, with a 3.65-fold change (*p* < 0.05), but F1 had no discernible effect on CYP1B1 mRNA expression. However, quercetin failed to modify CYP2S1 mRNA expression in MDA-MB-231 cells following 72 h of treatment. In contrast, F1 increased CYP2S1 mRNA expression in MDA-MB-231 cells at 24 h (1.80-fold change; *p* < 0.05) and 48 h (2.85-fold change; *p* < 0.001) of treatment (Figure 6(c)), which is consistent to the cytotoxic effect of F1 determined. However, no significant induction of CYP2S1 mRNA expression was observed at 72 h of F1 treatment. In comparison, MDA-MB-231 cells treated with F1 and quercetin for 72 h showed different mRNA expression levels of CYP1A1, CYP1B1, and CYP2S1 in the treated cells.

## 4. Discussion

The preliminary results of this study indicate the presence of quercetin in subfraction F1 and the standardized value of F1 derived from our research. The results then demonstrated the growth inhibitory activity of F1 (plant substance) and quercetin (pure compound), whereby F1 is better suited for treatments that require immediate effect, while quercetin could be used for long-term treatment. F1 induced cell cycle arrest at both the S and G2/M phases, but quercetin only induced cell cycle arrest at the S phase in MDA-MB-231 cells. Quercetin induced apoptosis in MDA-MB-231 cells, but F1 did not. The BrdU incorporation of DNA synthesis in MDA-MB-231 cells was not fully inhibited by 50 *µ*g/mL F1 and 60 *µ*g/mL quercetin at 24 and 48 h of treatment. F1 showed lower mRNA expression levels of CYP1A1 and CYP1B1 (procarcinogenic compounds metabolism) than quercetin, but a higher mRNA expression level of CYP2S1 (cytotoxicity) was found in F1-treated MDA-MB-231 cells than in quercetin-treated MDA-MB-231 cells for 72 h of treatment.

F1 was revealed to be a potential agent to exhibit an antiproliferative effect and cell cycle arrest in MDA-MB-231 breast cancer because F1 contains a significant amount of total flavonoid content and quercetin. F1 has a consistent absorption pattern, which directly proves the total flavonoid content and quercetin content in F1. This phenomenon also clearly indicates that the method used to obtain F1 is standardized, whereby F1 always shows a maximum absorption peak at 420 nm at a high concentration. The method used to obtain F1 also shows that most of the flavonols are retained during the dialysis fractionation process. Ethanol was more suitable for extracting polyphenolic compounds found in onion than methanol, ethyl acetate, chloroform, and acetone because ethanol is the most common solvent in laboratory settings, relatively safer, and less costly than other extraction solvents [18, 19]. This phenomenon strengthens the usage of ethanol as the extraction solvent to separate bioactive compounds in onion peels, such as anthocyanins, quercetin, and other flavonols, from the crude ethanolic extract of red onion peels (E1) [20, 21].

MDA-MB-231, a poorly differentiated, highly aggressive, and invasive breast cancer cell line, is a model representing triple-negative breast cancer, characterized by the lack of oestrogen receptor, progesterone receptor, E-cadherin, and HER2 growth factor receptor but presenting with mutated p53 gene expression [22, 23]. Therefore, MDA-MB-231 cells are the ideal cell model for investigating the effectiveness of newly developed chemotherapeutic agents. In this study, F1 and quercetin were found to reduce the proliferation of MDA-MB-231 cells by inducing different cell cycle arrest profiles. Regulation of the cell cycle is crucial for the development of healthy cells. Nevertheless, cancerous cells exhibit uncontrolled cell proliferation and evasion of apoptosis resulting from dysfunction of the cell cycle checkpoint and destruction [24]. Uncontrolled cell growth and apoptosis resistance are the major defects in cancer cells, thus, discovering potential compounds targeting cell cycle mechanisms and apoptotic machinery could be effective against uncontrolled cell proliferation.

F1 and quercetin were found to exhibit different cell cycle arrest profiles in MDA-MB-231 cells, suggesting different comprehensive effects of F1 and quercetin in MDA-MB-231 cells. One possible explanation is the presence of different compound compositions in F1, which gives rise to different molecular mechanisms of cell cycle regulation induced by F1. A study reported that 20 *µ*M quercetin induced cell cycle arrest at the S and G2/M phases in MDA-MB-231 cells after 48 h of treatment [25]. This finding was linked to the increased signalling activities of p21 and GADD45, which contributed to G1/S phase and G2/M phase arrest, respectively, regulated by p53. Another study indicated that cell cycle arrest was observed at the G2/M phase after treatment of MDA-MB-231 cells with 100 *µ*M quercetin for 24 and 48 h [16]. Nevertheless, Rivera's study showed cell cycle arrest at the G2/M phase in MDA-MB-231 cells after 48 h of treatment with 15 *µ*M quercetin [26]. In this study, cell cycle arrest was observed at the S phase only after treatment with 60 *µ*g/mL quercetin for 48 h, which is slightly in contrast to previously published findings, whereas F1 is able to obstruct cell cycle progression in both the S and G2/M phases. This difference may be due to variation in the cell treatment concentration, where a higher concentration of quercetin was utilized for the experiments. Apoptosis analysis showed that an apoptotic effect was observed in MDA-MB-231 cells treated with quercetin, but F1 did not induce apoptosis in MDA-MB-231 cells. The induction of apoptotic effects in MBA-MD-231 cells in this study was consistent with other findings using the same cell line [16, 25–27]. This result suggests that cell proliferation inhibition by F1 in MDA-MB-231 cells occurred through mechanisms other than the apoptosis pathway.

The F1 effect was further validated by detecting the proliferative cells incorporated with DNA synthesis using BrdU staining, where the dye acts as a thymidine analogue to replace thymidine nucleotides in the newly synthesized DNA [28]. The analysis found that a low percentage of BrdU-positive cells was detected in MDA-MB-231 cells treated with 50 *µ*g/mL F1 and 60 *µ*g/mL quercetin for 72 h. This phenomenon suggests that F1 inhibits DNA synthesis during cell proliferation only after 72 h of treatment. New cellular DNA content was still synthesized in MDA-MB-231 cells even after treatment with 50 *µ*g/mL F1 and 60 *µ*g/mL quercetin for 24 and 48 h. The decrease in cell viability observed in the cells that were treated with this F1 concentration and these treatment durations may be due to the toxicity derived from other bioactive compounds in F1, rather than the decrease in cellular DNA content.

CYP genes have been extensively confirmed to be involved in the metabolism of procarcinogenic compounds to highly carcinogenic metabolites [29, 30]. Other studies have shown that the genes encoding these proteins are linked to cell signalling pathways critical for cell cycle regulation [31]. For instance, the aryl hydrocarbon receptor (AHR) responsible for activating CYP gene transcription is a protein that affects cell cycle regulation [32]. Several findings have shown that dietary flavonoids play a role as AHR ligands with either antagonist or agonist activity to inhibit cancer cell growth [33–35]. Additionally, flavonoids may also undergo CYP1-mediated oxidative metabolism to become antiproliferative products [33]. A study demonstrated the antiproliferative and cytostatic effects of a flavonoid lipid molecule, eupatorine, in breast cancer cells due to the involvement of CYP1-mediated metabolism [36]. The studies showed that cell cycle arrest at the G2/M phase induced by eupatorine could be reversed when MDA-MB-468 cells were coincubated with the CYP1 inhibitor acacetin. Another finding by Atherton confirmed that metabolites produced from the isoflavones daidzein and genistein via CYP1A1, CYP1A2, and CYP1B1 metabolism induced an antiproliferative response in MCF-7 cells [37].

In this study, the analysis of CYP genes showed that F1 and quercetin induced mRNA expression of CYP1A1 and CYP1B1, with the highest level observed at 48 h of treatment. This phenomenon corresponded to the initiation of cell cycle arrest at the S phase by F1 and quercetin in MDA-MB-231 cells and the profound changes in cell cycle progression, which was also observed at 48 h of treatment with further induction of cell cycle arrest at the G2/M phase by F1. This finding is supported by numerous studies that revealed the role of quercetin in cancer proliferation in relation to its interaction with CYP family enzymes. For instance, quercetin was shown to be an agonist of CYP1A1 in breast cancer cells [38]. A study by Ciolino also showed that quercetin increases CYP1A1 mRNA level through mediation by the AHR receptor [39]. Furthermore, the metabolism of quercetin by the CYP1 enzyme, particularly CYP1A1 and CYP1B1, intensifies their antiproliferative effects in breast cancer cells [38]. Although F1 may not be as effective as quercetin in promoting metabolic activity, the results suggested that the antiproliferative effect of F1 and quercetin on MDA-MB-231 cells might be due to the metabolic activity of these CYPs, resulting in the production of active metabolites, which indirectly modulate the cell cycle progression and survival of MDA-MB-231 cells. For CYP2S1 gene expression analysis, F1 (but not quercetin) induced significantly high gene expression levels in MDA-MB-231 cells at 24 and 48 h of treatment. The selective expression of CYP2S1 in MDA-MB-231 cells treated with F1 suggested that CYP2S1 likely plays a role in the regulation of F1 anticancer activity, which is likely regulated by AHR [40].

In conclusion, the results provide more detailed information on the composition of the standardized subfraction F1, including its growth inhibitory activity, cell cycle arrest profile, and apoptosis induction in MDA-MB-231 cells in different ways. Moreover, inhibition of new cellular DNA synthesis and CYP gene expression may imply that F1 is a potential anticancer agent derived from the green approach towards breast cancer treatment.

## Figures and Tables

**Figure 1:** Ultra-performance liquid chromatography (UPLC), 360 nm of phenolic compounds. (a) F1 (1 mg/mL; isolated from batch 1 of red onion peel), (b) F1 (1 mg/mL; isolated from batch 2 of red onion peel), (c) quercetin (200 *μ*g/mL; standard), and (d) a standard curve of quercetin in the concentration range of 25 to 200 *μ*g/mL. Quercetin was dissolved in 99.7% ethanol.

**Figure 2:** Dose-response curves of MDA-MB-231 following treatments with F1 for (a) 24 h, (b) 48 h, and (c) 72 h and with quercetin for (d) 24 h, (e) 48 h, and (f) 72 h. The maximal response (inhibition rate at the maximum dose concentration) identified hillslope value (slope at EC_50_ value) and an EC_50_ value of each test compound from the curve. The experiments were repeated several times to ensure the repeatability and reproducibility of the results. All values are expressed as the means ± SD.

**Figure 3:** Flow cytometry of treated MDA-MB-231 cells on cell cycle after 72 h treatment. (a) Histograms of the cell cycle distribution of MDA-MB-231 cells after treatment by flow cytometry. (A) MDA-MB-231 was treated with 0.1% DMSO for 24 h (control), (B) DMSO-treated for 48 h, (C) DMSO-treated for 72 h, (D) 50 *μ*g/mL F1-treated for 24 h, (E) 50 *μ*g/mL F1-treated for 48 h, (F) 50 *μ*g/mL F1-treated for 72 h, (G) 60 *μ*g/mL quercetin-treated for 24 h, (H) 60 *μ*g/mL quercetin-treated for 48 h, and (I) 60 *μ*g/mL quercetin-treated for 72 h. The vertical (*y*) axis represents cell number, whereas the horizontal (*x*) axis represents a channel. (b) Analyzed cell cycle profile of F1 (50 *μ*g/mL) and quercetin (60 *μ*g/mL) in MDA-MB-231 cells after (A) 24 h, (B) 48 h, and (C) 72 h of treatment. Each dataset represents the mean of two independent experiments with triplicate readings each. Significant differences were analyzed versus control using one-way ANOVA and Dunnett's multiple comparison test indicated as ^*∗*^*P* < 0.05; ^*∗∗*^*P*<0.01; and ^*∗∗∗*^*P*<0.001. Control: DMSO-treated cells.

**Figure 4:** Flow cytometry of treated MDA-MB-231 apoptotic and necrotic cells after 72 h treatment. (a) Histograms of the apoptotic and necrotic distribution of MDA-MB-231 cells after treatment by flow cytometry. (A) MDA-MB-231 was treated with 0.1% DMSO for 24 h (control), (B) DMSO-treated for 48 h, (C) DMSO-treated for 72 h, (D) 50 *μ*g/mL F1-treated for 24 h, (E) 50 *μ*g/mL F1-treated for 48 h, (F) 50 *µ*g/mL F1-treated for 72 h, (G) 60 *μ*g/mL quercetin-treated for 24 h, (H) 60 *μ*g/mL quercetin-treated for 48 h, and (I) 60 *μ*g/mL quercetin-treated for 72 h. After staining with FITC-conjugated annexin and propidium iodide, the flow cytometer analyzed the cells. The lower left and upper left quadrants represent the percentage of viable and necrotic cells. In contrast, the early and late apoptosis events are shown in the lower and upper right quadrants. (b) Analyzed apoptotic and necrotic profiles of F1 (50 *μ*g/mL) and quercetin (60 *μ*g/mL) in MDA-MB-231 cells after (A) 24 h, (B) 48 h, and (C) 72 h of treatment. Each dataset represents the mean of two independent experiments with triplicate readings each. One-way ANOVA and Dunnett's multiple comparison test were used to interpret statistically significant differences between treated and untreated cells (control) as ^*∗*^*P* < 0.05 and ^*∗∗∗*^*P*<0.001. EA: early apoptosis, LA: late apoptosis.

**Figure 5:** Flow cytometry of BrdU-positive treated MDA-MB-231 cells after 72 h treatment. (a) Representative dot-plot analysis showing the proportion of BrdU-positive treated MDA-MB-231 cells by flow cytometry. (A) MDA-MB-231 cells were treated with 0.1% DMSO for 24 h (control), (B) DMSO-treated for 48 h, (C) DMSO-treated for 72 h, (D) 50 *µ*g/mL F1-treated for 24 h, (E) 50 *μ*g/mL F1-treated for 48 h, (F) 50 *μ*g/mL F1-treated for 72 h, (G) 60 *µ*g/mL quercetin-treated for 24 h, (H) 60 *μ*g/mL quercetin-treated for 48 h, and (I) 60 *μ*g/mL quercetin-treated for 72 h. The cells enclosed in the box gate labelled with R6 were used to calculate the percentage of BrdU-positive cells. (b) Percentage of BrdU-positive treated MDA-MB-231 cells. The percentage of BrdU-positive MDA-MB-231 cells treated with 0.1% DMSO (control), 50 *μ*g/mL F1, and 60 *μ*g/mL quercetin was determined by flow cytometry. The bar chart represents the mean ± SD of two independent experiments with significant differences indicated as ^*∗*^*P* < 0.05, ^*∗∗*^*P*<0.01, and ^*∗∗∗*^*P*<0.001 compared to the controls. One-way ANOVA and Dunnett's multiple comparison test were used for the statistical analysis.

**Figure 6:** Effect of F1 (50 *μ*g/mL) and quercetin (60 *μ*g/mL) on the mRNA gene expression of (a) CYP1A1, (b) CYP1B1, and (c) CYP2S1 in MDA-MB-231 cells. The mRNA expression was normalized to the expression of GAPDH in each sample. The bar chart represents the mean ± SD of two independent experiments with significant differences indicated as ^*∗*^*P* < 0.05, ^*∗∗*^*P*<0.01, and ^*∗∗∗*^*P*<0.001, compared to the controls. One-way ANOVA and Dunnett's multiple comparison test were used for the statistical analysis.

**Table 1:** The list of primers used for real-time PCR.

Gene	Primer sequence	Size amplicon
CYP1A1	Forward 5′-TCAGGAGAAGCAGCTGGATGA-3′	76 bp
	Reverse 5′-GAGGTCCAAGACGATGTTAATGATC-3′	

CYP1B1	Forward 5′-ATCAGGTGAGGTGTGCTCCAT-3′	70 bp
	Reverse 5′-TCTCCCAGAAGCTCCTGCATA-3′	

CYP2S1	Forward 5′-GACAGGGTTAATGTCTCCAGAGTGT-3′	78 bp
	Reverse 5′-GGACAGACTCCGGAAAACAACT-3′	

GAPDH	Forward 5′-ACAGCCTCAAGATCATCAGCA-3′	137 bp
	Reverse 5′-AGTCTTCTGGGTGGCAGTGAT-3′	

## Data Availability

No specific datasets were used and/or analyzed during this study. The datasets are available from the corresponding author and can be presented at reasonable request.
